# Chronic Kidney Disease and Calciphylaxis: A Literature Review

**DOI:** 10.7759/cureus.3334

**Published:** 2018-09-19

**Authors:** Munis M Ahmed, Asma Zakir, Muhammad Farhan Ahsraf, Amna Ejaz, Aqsa Ashraf, Lalith Namburu, Muhammad S Farooqi, Moeed Ahmed, Ibrahim Raza

**Affiliations:** 1 Internal Medicine, King Edward Medical University, Mayo Hospital, Lahore, PAK; 2 Internal Medicine, Siddhartha Medical College, Vijayawada, IND

**Keywords:** chronic kidney disease (ckd), kidney, calciphylaxis, chronic

## Abstract

Calcific uremic arteriolopathy (CUA), also known as calciphylaxis, is a rare complication of chronic kidney disease (CKD). Its incidence is increasing due to a better understanding and diagnosis by physicians. Calciphylaxis is a fatal complication of many metabolic disorders. If not managed properly, it can lead to death within a year. This review is an effort to highlight the importance of research on prompt diagnosis and treatment guidelines for calciphylaxis, as it poses a challenge due to its diverse clinical presentation and high mortality rate.

## Introduction and background

Calcific uremic arteriolopathy (CUA), also known as calciphylaxis, is a rare complication of chronic kidney disease (CKD) where there is occlusion of microvasculature with mural calcification of the arterioles, causing severe ischemia and necrosis of the tissue [1]. CUA is a major condition presenting as the sequelae of many disorders. It is specified by the calcification of small vessels, especially arterioles, which subsequently lead to the obstruction of the blood flow. This obstruction causes ischemia, necrosis, severe pain, and color changes at the site. In this article, we discuss CUA as a major complication of CKD. Its importance lies in the fact that it is a "fatal" disease with a huge chance of further complications, leading to increased morbidity and mortality. Its presentation may also be diverse, thus posing a great challenge for the practitioners to separate and identify it among the possibility of other, more widely known differentials. Moreover, its incidence is increasing day by day, emphasizing the need for extensive research and awareness among the medical community in order to diagnose and treat it on a timely basis. If not diagnosed and managed on time, the patient’s condition can deteriorate very fast. In this review, we discuss the multiple presentations reported across a widespread area. We will also discuss the diagnostic tools, standardized methods in comparison to the practical, clinical bedside approach, their efficacy and efficiency in obtaining prompt results and diagnosis, and lower risk factors without further exacerbating the patient’s condition. We will also emphasize the importance of different management options available at the moment and how to manage a patient timely and properly and to consider less practiced options according to the clinical situation and requirement of the patient, in order to save his/her life. Our main aim is to highlight this major issue and to stress upon its importance so that lives can be saved.

Bryant and White first explained the rare condition of calcification and cutaneous necrosis in 1898 [2]. Its pathophysiology was highlighted for the first time by Selye et al. They named the disease in 1962 and concluded that it is a systemic hypersensitivity reaction. They then conducted several animal studies where they could experimentally prove the induction of calcification of many organs by exposing them to various substances called sensitizing agents. The substances used were vitamins D2 and D3, parathyroid hormone (PTH), and dihydrotachysterol. They were exposed to challenging situations, such as trauma or metallic ions (iron, aluminum). Ketteler et al [3-5]. inferred that calcification can cause a disturbance of two Vitamin K-dependent calcification inhibiting proteins known as Matrix-Gla and Fetuin-A [6]. It was further proved by animal experimentation that a deficiency of these proteins can cause a calcification of arteries and the subsequent rupture of major arteries like the aorta [7-8].

Calcific uremic arteriolopathy (CUA) is characterized by obstructive vasculopathy, where small arteries and arterioles are calcified. This calcification results in the narrowing of the lumen, causing occlusion and subsequent ischemia and cutaneous necrosis. It is typically found in patients with end-stage renal failure (ESRF). Its incidence in patients on hemodialysis is 1% to 4% [9]. Some sporadic instances have also been reported, where calciphylaxis presents with normal renal function [10]. Recent recipients of a renal transplant may also present with CUA [11]. Mortality associated with calciphylaxis is high, with an estimated one-year rate of survival of 45%-80% [12-13].

In addition to kidney failure, other risk factors causing CUA include obesity, female sex, white race, liver disease, elevated calcium-phosphorus products, medications (warfarin, systemic steroids, calcium binders, and vitamin D analogs), a hypercoagulable state, and hypoalbuminemia. Warfarin is most frequently associated with the disease [10,14-16]. Parathyroid hormone is often found to be abnormal. In previously reported cases, 76% of patients with penile necrosis secondary to calcific uremic arteriolopathy have concurrent diabetes as compared to 39% of ESRF patients, which suggests that diabetes is also a major predisposing factor in the development of penile CUA [17].

## Review

Calcific uremic arteriolopathy (CUA) has a multifactorial pathogenesis. The main pathophysiology of CUA is where inducers and inhibitors of calcification in the vascular wall are in a state of imbalance. Conversion of vascular smooth muscle into osteoblast-like-cells is encouraged by elevated serum phosphate levels, thus encouraging vascular calcification. Moreover, uremia resulting from end-stage renal failure (ESRF) causes the enhanced suppression of calcification inhibitors by creating an inflammatory reaction.

All this leads to vascular calcification, thrombosis, luminal narrowing, ischemia, and skin necrosis. First of all, a primary lesion is formed when calcium salts accumulate in the media of small arteries, causing the narrowing of the arterial lumen. As a result, there is a diminished arteriolar blood flow, which leads to ischemia, subsequently causing pain. If the ischemia is long enough, necrosis develops. Lesions develop in areas where there is a lot of adipose tissue. Excess weight causes excessive stress on dermal arterioles that are responsible for focally dystrophic calcifications [18-19]. Primary lesions are not clinically manifested but rather seen upon radiological imaging. Secondary lesions, which consist of the infarcts, are seen in the soft tissues.

Clinical presentation

Calciphylaxis can clinically manifest in two phases. The first phase presents with pruritus and cutaneous laminar erythema, presenting as a violaceous rash, which is nonspecific and may resemble livedo reticularis. Therefore, in this stage, misinterpretation can easily be made. The second phase presents with a rash that progresses to painful eschars and later develops into painful non-healing ulceration and necrosis [20]. The most common involvement is of the lower extremities. Arteriolar medial calcification and fat tissue are particular to CUA and mainly affect the skin but, in some instances, other organs like nerve sheaths, visceral organs, and muscles may also be involved. In penile calcific uremic arteriolopathy, two-thirds of the patients have gangrenous lesions on extragenital areas [17]. This emphasizes that that calcifications are often extensive and widespread throughout the body. The main differential diagnoses include pyoderma gangrenosum, coagulopathies, and arteriosclerotic ulcers.

Diagnosis

CUA is a major complication of CKD, which demands timely diagnosis. It carries a high risk of mortality and various complications. So, if not diagnosed on time, it can lead to serious ramifications for the patients and a major decrease in the prognosis. A “skin biopsy” is considered to be the standardized diagnostic test. But clinically, it is often not the first choice due to the high risk of poor healing or non-healing and the resulting infection [21]. It can also cause sepsis and necrotic spread, leading to a deterioration in the condition [22]. Hence, the ideal criteria for the diagnosis are the clinical presentation, metabolic parameters, and radiological findings. The findings obtained on imaging are very specific and usually show the calcification of tunica media of the arterioles. Smaller subcutaneous vessels also show calcification [23]. A potential metabolic indicator for diagnosis is a calcium phosphate product over 70 mg/dL [17]. It has also been observed that penile calcific uremic arteriolopathy had a significantly higher calcium phosphate product than a control group of patients with ESRF (p < 0.05).

Management

After the diagnosis, proper management and treatment play a vital role in decreasing the suffering of the patient, avoiding further complications and lowering the mortality rate to some degree. Even after all the possible measures, the overall fatality rates remain high. But this should not deter us from looking for better options of management. The standard therapeutic options include pain management, conservative therapy, and surgical management. First-line conservative measures include aggressive wound care (debridement, incision drainage), systemic antibiotics, aggressively managing the renal disease with daily hemodialysis, non-calcium containing phosphate binders, cinacalcet (a calcium-receptor stimulating agent), bisphosphonates, and, the most promising of all, sodium thiosulfate.

Cinacalcet is a calcimimetic agent. It makes the parathyroid gland more sensitive to calcium, hence, it acts to inhibit PTH release. Cinacalcet use in calciphylaxis, as shown in many case reports, accelerates wound healing [24].

Sodium thiosulfate has a major and vital role in the treatment of calcific uremic arteriolopathy. Its use shows marked improvement after just two weeks. After continuous use for eight months, it is said to completely resolve the pain [25]. Sodium thiosulfate acts by converting insoluble calcium in the tissues to soluble calcium thiosulfate [26], thus improving the solubility of the calcium deposits and facilitating the removal of these deposits by mobilizing them. It also has antioxidant properties that protect against any reactive oxygen species or inflammatory products, thus preserving the wall integrity [27-28]. It causes the increased formation of endothelial nitric oxide that dilates the vessels and improves the circulation decreasing ischemia [29].

Surgery is not a favored line of treatment for these patients. Surgical stress can result in increased excitation of the sympathetic nervous system. This can cause a disruption in circulation and widespread necrosis [22]. Due to these problems, surgery is limited and generally indicated for patients with intractable pain, after the patient shows no response to the conservative therapy.

Diverse patterns of vascular calcification

Vascular calcification shows diverse patterns on plain radiographs: Intimal calcification is thought to appear as a patchy or irregular pattern or medial calcification may appear as a linear or railroad-track arrangement. Calciphylaxis has been traditionally associated with linear calcification. But recently, a case report was presented in Florida in which end-stage renal disease (ESRD) patients with calciphylaxis and extensive vascular calcifications patterns were reported [30]. Three ESRD patients presented with lower extremity lesions that were consistent with CUA findings. Upon examination, all three showed distinct patterns of vascular calcification. The first patient had a serum parathyroid hormone (PTH) of 849 pg/mL (150–300 pg/ml for ESRD). On imaging, “linear calcifications” were seen. The patient was given sodium thiosulfate therapy, which is currently the standard treatment, in addition to the intensification of the dialysis regimen and the optimization of serum calcium and phosphate levels. The patient showed promising improvement [31]. The second patient had a PTH level of 1099 pg/mL. The radiological studies showed “patchy vascular and soft tissue calcifications,” and this patient also improved with the administration of sodium thiosulfate. The third patient with a PTH level of 553 pg/mL had calcifications with a “railroad-track appearance.” But the sodium thiosulfate therapy didn’t work because infection and gangrene had already set in. So amputation was required to save the patient’s life. All three patients were in their fifties and had increased phosphate levels and a long history of dialysis. This shows that the pattern of calcification may vary from person to person, and CUA alone can show diversity in the calcification pattern. However, the ultimate treatment plan and prognosis depends upon the clinical symptoms and complications of the disease at the time of presentation and even after the start of the therapy.

Calcific uremic arteriolopathy presenting with penile lesion

A case was reported by NHS in London, UK, where a patient with ESRF came to the emergency room (ER) with the complaint of a solid, tender penile mass. A sample of the excised lesion was sent for histopathological analysis. Microscopic findings were consistent with the findings of CUA showing tissue necrosis, vascular calcification leading to luminal narrowing, hyperplasia of the tunica intima, and infiltration of the tissue with inflammatory cells. No evidence of malignancy was found. Immediately after the operation, there were no complications. So the patient was referred for the management of his renal disease. But late complications developed due to a poor healing of the wound. The condition of the patient deteriorated with widespread sepsis. The patient died after one month of surgery [32].

Calciphylaxis in a pediatric patient

Calciphylaxis has a relatively low incidence in the pediatric age group. But it must not be ruled out in patients with positive risk factors [33]. A case report from National Health Service (NHS), Liverpool, UK, reported a 17-year-old who suffered a small injury on the dorsum of his right foot. It developed into a painful, erythematous lesion. On examination, the lesion was approx 0.5 cm in diameter, cold to touch, with a well-formed edge around widespread petechiae. The intensity of the pain made his foot immobile and unable to bear weight. The patient had immunoglobulin A (IgA) nephropathy that had progressed to CKD stage five and had been receiving treatment in the form of hemodialysis for 16 months. Serum calcium, phosphate, and parathyroid hormone (PTH) were abnormally raised. The patient was non-compliant with both medication and diet. Based on this clinical picture, calciphylaxis was diagnosed. A new treatment plan was formulated. The patient underwent daily dialysis, and vitamin D analogs and calcium-based phosphate binders were ceased. Cinacalcet was initiated. Opiate analgesia was administered to tackle severe pain. Hence, with the control of the calcium phosphate product, the overall condition of the lesion and the patient improved tremendously [34].

Role of urgent parathyroidectomy in calciphylaxis

A case report from Patras University School of Medicine showed a patient on continuous ambulatory peritoneal dialysis (CAPD) who was completely nonresponsive to medical treatment and presented with severe complications of calciphylaxis [35]. The patient did not respond to any treatment. To prevent the deteriorating condition of the patient, an urgent parathyroidectomy was performed. Post-operatively, the calcium phosphate product and the physical condition of the patient was monitored closely. Great results were seen, as there was a significant drop in the calcium-phosphate product. Also, the skin lesions and physical well being of the patient was improved dramatically. The patient was discharged with excellent recovery. Hence, it is generally acceptable to perform urgent parathyroidectomy to treat this disorder considering the clinical picture after medical therapy has failed. But no definite conclusions can be made, as series reports usually have a limited number of patients and show a selection bias [36-37].

## Conclusions

Calcific uremic arteriolopathy was considered a rare diagnosis but not anymore. It is being increasingly reported with an increasing number of patients with chronic kidney disease. The early identification of risk factors and diagnosis acquires center stage in improving the outcome for patients. If the condition is detected early, there is a better chance of managing the symptoms and improving the quality of life for the patient. Though relatively rare, chronic kidney disease in children can lead to calciphylaxis. Despite major efforts for early diagnosis, prompt therapy, and revolutions in the management drugs, the fact remains that calciphylaxis in chronic kidney disease is still a severe complication that more often than not leads to death.
